This article has been retracted.

# Long non-coding RNA SNHG14 exerts oncogenic functions in non-small cell lung cancer through acting as an *miR-340* sponge

**DOI:** 10.1042/BSR20180941

**Published:** 2019-01-03

**Authors:** Zhenhua Zhang, Yong Wang, Wei Zhang, Junyan Li, Weiliang Liu, Wenming Lu

**Affiliations:** 1 Department of Cardiothoracic Surgery, 3201 Hospital of Hanzhong City, Shaanxi Province 723000, China; 2 Department of General Surgery, The People’s Hospital of Nanzheng County, Shaanxi Province 723100, China

**Keywords:** cell cycle, long non-coding RNA, miR-340, non-small cell lung cancer, prognosis, SNHG14

## Abstract

Long non-coding RNA (lncRNA) SNHG14 is previously found to be overexpressed in several types of cancers. However, the clinical significance and biological function of SNHG14 in non-small cell lung cancer (NSCLC) are still elusive. In the present study, we found that SNHG14 was aberrantly up-regulated in NSCLC tissues from patients and cell lines compared with their normal counterparts. Increased SNHG14 expression was closely associated with aggressive tumor progression and poor clinical outcome of NSCLC patients. Knockdown of SNHG14 inhibited NSCLC cell proliferation through inducing cell cycle arrest and apoptosis, whereas SNHG14 overexpression exerted the opposite effects. Animal experiment further revealed that down-regulated SNHG14 greatly inhibited NSCLC tumor growth *in vivo*. Further studies demonstrated that SNHG14 might serve as a competing endogenous RNA (ceRNA) by sponging *miR-340* in NSCLC cells. Taken together, our study demonstrated that SNHG14/*miR-340* axis might play a novel role in regulating the malignant behaviors of NSCLC, which provided a new potential diagnostic and therapeutic strategy for this malignant disease.

## Introduction

Lung cancer is the leading cause of cancer-related deaths worldwide, which is a serious threat to human health [1]. Amongst all lung cancer cases, non-small cell lung cancer (NSCLC) accounts for approximately 85%, and adenocarcinoma is one of the main histological types [2]. Despite great advances in therapeutic methods, the prognosis of NSCLC patients remains dismal, with the 5-year survival rate of less than 15% [3]. Thus, it is of great importance to explain the molecular mechanisms underlying the initiation and progression of NSCLC, and identify novel therapeutic targets to improve the efficacy of clinical anti-NSCLC management.

The human genome expresses tens of thousands of long non-coding RNAs (lncRNAs), which are a type of RNA molecules greater than 200 nts in length with little protein-coding potential [4,5]. LncRNAs are often expressed in a spatial- and temporal-specific pattern [4]. Recent studies revealed that lncRNAs can function as an oncogene or tumor suppressor in a variety of cancer types, including NSCLC [6,7]. In this regard, highlighting the potentially widespread functional roles of lncRNAs in NSCLC is of critical importance.

Small nucleolar RNA host gene 14 (SNHG14), a novel lncRNA mapping to 15q11.2 in humans, was previously shown to be overexpressed and exert its oncogenic activity in various human malignancies, including clear cell renal cell carcinoma [8] and gastric cancer [9]. However, as far as we know, there is limited research that discloses the functional role of SNHG14 in the development of NSCLC.

In the current study, we explored the clinical feature, biological function, and potential mechanism of SNHG14 in NSCLC. We believed that our findings might provide a novel diagnostic predictor and a valuable therapeutic target for NSCLC in the future.

## Materials and methods

### Patients and tissue samples

Paired NSCLC tissues and adjacent normal lung tissues were collected from 99 cases of patients, who underwent surgical resection at 3201 Hospital of Hanzhong City (Shaanxi, China). Patients who received chemotherapy or radiotherapy prior to surgery were excluded in this study. All tissue specimens were immediately snap-frozen in liquid nitrogen and stored at −80°C until further use. All tumor and paired normal tissues were verified by experienced pathologists. The clinicopathological characteristics of these patients were listed in Table 1. Overall survival (OS) was defined as the interval between resection and death or the last follow-up visit. Our study was approved by the Ethics Committee of 3201 Hospital of Hanzhong City, and written informed consents were obtained from all participants.

**Table 1:** Correlation between SNHG14 expression and clinicopathological features of NSCLC patients

Characteristics	Total number	SNHG14 expression		*P*-value
		Low (*n*=56)	High (*n*=43)	
Age				0.421
<65	39	24	15	
≥65	60	32	28	
Gender				0.839
Male	68	38	30	
Female	31	18	13	
Smoking history				0.212
Nonsmoker	73	44	29	
Ever-smoker	26	12	14	
Tumor location				0.853
Left lung	54	31	23	
Right lung	45	25	20	
Histology type				0.132
Adenocarcinoma	50	32	18	
Squamous	49	24	25	
Tumor size				0.047
<5 cm	68	43	25	
≥5 cm	31	13	18	
Lymph node metastasis				0.061
No	61	39	22	
Yes	38	17	21	
TNM stage				0.046
I	47	31	16	
II	29	17	12	
III + IV	23	8	15	

### Cell culture and transfection

The human NSCLC cells A549, NCI-H1975, NCI-H1299, SK-MES-1 and normal human bronchial epithelial 16HBE cells, obtained from the Institute of Biochemistry and Cell Biology at the Chinese Academy of Sciences (Shanghai, China), were cultured in the RPMI 1640 medium (KeyGene, Nanjing, China) containing 10% FBS (Invitrogen, Carlsbad, CA, U.S.A.) and antibiotics (100 U/ml penicillin and 100 mg/ml streptomycin) at 37 °C in an atmosphere containing 5% CO_2_.

Human *miR-340* mimics and corresponding mimics control were purchased from GenePharma (Shanghai, China). The sequences of three siRNAs specifically targetting SNHG14 (si-SNHG14) and a scrambled nucleotide (si-NC) were listed as follows: si-SNHG14-1: 5′-CAGCAUAUGUAAGUGGAACUCAGAA-3GC si-SNHG14-2: 5′-GCAAUCAUGACUGUUGGCAAGAGUA-3′, si-SNHG14-3: 5′-GGCCGAAUCUUCAUUGGCACCUUUA-3CCGAAUCUUCAUUGGCACCGAACGUGUCACGUUU-3′. The full-length human SNHG14 sequence was amplified by PCR, and the PCR product was subcloned into a pcDNA3.1 vector (Invitrogen) and named pcDNA3.1-SNHG14. A scrambled negative control (pcDNA3.1-NC) was also constructed. Plasmids, siRNAs, *miR-340* mimics, and their negative controls were delivered to cells using Lipofectamine 2000 Reagent (Invitrogen). At 48 h post-transfection, cells were harvested and processed for further analysis. The sequence of shRNA against SNHG14 or scrambled control shRNA sequence was ligated into the pLKO.1-Puro vector (TaKaRa, Dalian, China) and then transfected into HEK293 cells. At 48 h after transfection, lentiviral particles were collected to infect A549 cells. A549 cells stably transfected with sh-SNHG14 or sh-NC were then screened with puromycin (10 μg/ml) for 2 weeks.

### RNA extraction, reverse transcription, and quantitative real-time PCR

Total RNA was extracted from prepared cell lines or tissues using TRizol reagent (Invitrogen). RNA concentration and quality were measured using a NanoDrop 2000 Spectrophotometer (Thermo Fisher Scientific, Inc., Waltham, MA, U.S.A.). For lncRNA quantitation, RNA was reverse transcribed to cDNA using PrimeScript RT reagent Kit (TaKaRa). For miRNA quantitation, reverse transcription was performed using OneStep PrimeScript miRNA cDNA Synthesis Kit (Qiagen, Valencia, CA, U.S.A.). After reverse transcription, qPCR analysis was performed using SYBR Premix ExTaq II Kit (TaKaRa) on ABI 7500 Real-time PCR System (Life Technologies, Carlsbad, CA, U.S.A.). GAPDH or U6 was used for the normalization of lncRNA and miRNA, respectively. Relative quantitation of tested gene expression was calculated and normalized by the 2^−ΔΔ*Ct*^ method [10]. The sequences of primers used here were listed in Table 2.

**Table 2:** The sequences of the primers

Gene name	Primer sequences
*SNHG14* forward primer	5′-GGGTGTTTACGTAGACCAGAACC-3′
*SNHG14* reverse primer	5′-CTTCCAAAAGCCTTCTGCCTTAG-3′
*GAPDH* forward primer	5′-CGAGATCCCTCCAAAATCAA-3′
*GAPDH* reverse primer	5′-TTCACACCCATGACGAACAT-3′
*miR-340*-RT	5′-GTCGTATCCAGTGCAGGGTCCGAGGTATTCGCACTGGATACGACAATCAG-3′
*miR-340* forward primer	5′-TTATAAAGCAATGAGA-3′
*miR-340* reverse primer	5′-GTGCAGGGTCCGAGGT-3′
*U6*-RT	5′-GTCGTATCCAGTGCAGGGTCCGAGGTATTCGCACTGGATACGACAAAATA-3′
*U6* forward primer	5′-CTCGCTTCGGCAGCACATATACT-3′
*U6* reverse primer	5′-ACGCTTCACGAATTTGCGTGTC-3′

### Cell proliferation assay

Cell proliferation was assessed using the Cell Counting Kit-8 (Dojindo, Tokyo, Japan). Briefly, after transfection, the cells were seeded (2 × 10^3^ cells/well) on six-well plates and cultured for 24, 48, 72, and 96 h, respectively. Twenty microliters of CCK8 solution was added to each well at indicated times. After an additional 2 h of incubation, the absorbance was measured at 450 nm using a microplate reader (Molecular Devices, Menlo Park, CA, U.S.A.).

### Cell cycle distribution analysis

For cell cycle analysis, the transfected cells were plated in six-well plates and further incubated for 48 h. Next, the cells were washed in PBS and fixed with 75% cold ethanol overnight, treated with RNase A, and then stained with propidium iodide using the Cycle TEST PLUS DNA Reagent Kit (BD Biosciences, San Diego, CA, U.S.A.). After incubation, the cells were subjected to flow cytometry analysis.

### Cell apoptosis analysis

For cell apoptosis assay, after transfection, cells were harvested, washed twice with cold PBS, and stained using the Annexin V-FITC apoptosis kit (Sigma–Aldrich Chemical Company, St. Louis, MO, U.S.A.). Subsequently, the percentage of apoptotic cells was analyzed by flow cytometry.

### Dual luciferase reporter assay

Full-length human SNHG14 fragment containing the predicted *miR-340*-binding site was cloned into the pLUC Luciferase vector (Ruibo, Guangzhou, China) and named pLUC-SNHG14-WT. A mutant reporter construct was created by using Quickchange XL Site-Directed Mutagenesis Kit (Agilent Technologies, Santa Clara, CA, U.S.A.) and named pLUC-SNHG14-MUT. A549 cells grown in 96-well plates were cotransfected with *miR-340* mimics or mimics control, pLUC-SNHG14-WT or pLUC-SNHG14-MUT, using Lipofectamine 2000 reagent. The luciferase activity was measured by using a luciferase reporter assay system (Promega, WI, U.S.A.) after 48 h of transfection.

### Xenograft experiment

Eight male athymic BALB/c nude mice (4–6 weeks old), obtained from the Animal Center of Shanghai Laboratory (Shanghai, China), were kept in a specific pathogen-free environment. A549 cells (2 × 10^6^) stably transfected with sh-SNHG14 or sh-NC were subcutaneously injected into the flanks of nude mice (*n*=4 per group). When the tumors were first grossly visible, the tumor volumes were measured every 3 days with a vernier caliper and calculated using the following formula: volume (mm^3^) = length × width^2^ × 0.5. After 19 days of cell injection, the mice were killed and the tumor weights were measured. The experiments were approved by the Ethics Committee of 3201 Hospital of Hanzhong City, and every effort was made to minimize animal suffering according to the NIH Guide for the Care and Use of Laboratory Animals [11].

### Statistical analysis

Statistical analyses were performed by SPSS 19.0 software package (IBM SPSS Inc; Chicago, IL, U.S.A.) and GraphPad Prism 6.0 (GraphPad Software Inc., CA, U.S.A.). Experimental data were presented as means ± S.D. of at least three independent experiments, and comparison between two groups was performed by two-tailed Student’s *t* test. The association between SNHG14 expression and clinicopathological features of NSCLC patients was evaluated using the Chi-square test. The OS of the patients was calculated with Kaplan–Meier method, and data were analyzed by the log-rank test. The correlation between SNHG14 and *miR-340* expression was evaluated by Pearson correlation analysis. *P*<0.05 was considered as significant difference.

## Results

### SNHG14 is up-regulated in NSCLC tissues and cell lines

To understand the biological significance of SNHG14 in NSCLC development, the levels of SNHG14 were examined in human NSCLC tissues and corresponding noncancerous tissues from 99 NSCLC patients using RT-qPCR analysis. The results showed that SNHG14 expression was significantly higher in cancer tissues compared with that in matched noncancerous tissues (Figure 1A). Meanwhile, we examined the correlation between SNHG14 expression and the clinicopathologic characteristics of 99 NSCLC patients. The patients were divided into the low expression group (<mean; *n*=56) and the high expression group (>mean; *n*=43), based on the median expression level of SNHG14 in all NSCLC tissues. As exhibited in Table 1, the high expression of SNHG14 in NSCLC was closely associated with larger tumor size (*P*=0.047) and advanced TNM stage (*P*=0.046). Kaplan–Meier analysis indicated that the prognosis was more unfavorable in NSCLC patients with high SNHG14 expression than those with low expression (*P*=0.04; Figure 1B). We next examined the expression of SNHG14 in a number of NSCLC cell lines, and observed that increased SNHG14 expression could be observed in all four NSCLC cell lines, compared with normal 16HBE cells (Figure 1C).

**Figure 1:** SNHG14 is up-regulated in NSCLC tissues and cell lines (**A**) SNHG14 expression was increased in NSCLC tissues compared with the adjacent nontumor tissues. (**B**) OS was compared between NSCLC patients with high SNHG14 expression and those with low SNHG14 expression. (**C**) SNHG14 expression was increased in a panel of NSCLC cells (A549, NCI-H1975, NCI-H1299, SK-MES-1) compared with normal 16HBE cells. Data were represented as the mean  ±  S.D. *P<0.05 compared with 16HBE cells.

### Knockdown of SNHG14 inhibits the proliferation of NSCLC cells

To further investigate the function of SNHG14 in NSCLC, we designed three siRNAs to knockdown SNHG14 in A549 cells (Figure 2A). si-SNHG14-2 was selected for further study. CCK-8 proliferation assay was performed to detect cell proliferation, and we found that the cell proliferation was suppressed significantly in si-SNHG14-transfected A549 cells (Figure 2B). Moreover, flow cytometry was used following transfection to assess cell cycle distribution and cell apoptosis. Compared with si-NC-transfected cells, knockdown of SNHG14 dramatically induced G_0_/G_1_ cell arrest in A549 cells (Figure 2C). Besides, knockdown of SNHG14 dramatically induced apoptosis of A549 cells (Figure 2D).

**Figure 2:** Knockdown of SNHG14 inhibits the proliferation of NSCLC cells (**A**) Validation of SNHG14 knockdown efficiency in A549 cells as determined by RT-qPCR analysis. (**B**) Cell proliferation was determined by CCK-8 assay in A549 cells transfected with si-SNHG14 or si-NC. (**C**) Cell cycle distribution was determined by flow cytometer analysis in A549 cells transfected with si-SNHG14 or si-NC. (**D**) Cell apoptosis was determined by flow cytometer analysis in A549 cells transfected with si-SNHG14 or si-NC. Data were represented as the mean  ±  S.D. *P<0.05 compared with si-NC group.

### Overexpression of SNHG14 promotes the proliferation of NSCLC cells

Overexpression of SNHG14 was successfully achieved through the transfection of pcDNA3.1-SNHG14 into A549 cells (Figure 3A). CCK-8 assay showed that the proliferation of A549 cells was significantly enhanced following SNHG14 overexpression (Figure 3B). We also determined the effects of SNHG14 overexpression on NSCLC cell cycle progression. The data showed that the cell population in the G_0_/G_1_ phase was reduced, whereas the S phase population was expanded after overexpression of SNHG14 (Figure 3C).

**Figure 3:** Overexpression of SNHG14 promotes the proliferation of NSCLC cells (**A**) Validation of SNHG14 overexpression efficiency in A549 cells as determined by RT-qPCR analysis. (**B**) Cell proliferation was determined by CCK-8 assay in A549 cells transfected with pcDNA3.1-SNHG14 or pcDNA3.1-NC. (**C**) Cell cycle distribution was determined by flow cytometer analysis in A549 cells transfected with pcDNA3.1-SNHG14 or pcDNA3.1-NC. Data were represented as the mean  ±  S.D. *P<0.05 compared with pcDNA3.1-NC group.

### Knockdown of SNHG14 inhibits NSCLC tumor growth *in vivo*

To validate whether SNHG14 regulates NSCLC cell proliferation *in vivo*, we established xenograft tumor models in nude mice using A549 cells transfected with sh-SNHG14 or sh-NC. As shown in Figure 4A, knockdown of SNHG14 significantly inhibited NSCLC tumor growth *in vivo*. Xenograft tumors derived from A549 cells transfected with sh-SNHG14 showed a smaller volume and lower weight than those derived from cells transfected with sh-NC (Figure 4B). Additionally, the down-regulation of SNHG14 in the tumors derived from sh-SNHG14-transfected A549 cells was confirmed by RT-qPCR analysis (Figure 4C).

**Figure 4:** Knockdown of SNHG14 inhibits NSCLC tumor growth *in vivo* (**A**) Growth curves of tumor volumes in different groups of nude mice. (**B**) At the experimental end point, tumors were dissected, weighted, and photographed. (**C**) RT-qPCR analysis of SNHG14 expression levels in the excised tumor tissues. Data were represented as the mean  ±  S.D. *P<0.05 compared with sh-NC group.

### SNHG14 acts as a sponge for *miR-340* in NSCLC cells

Through bioinformatics tool starBase v2.0 (http://starbase.sysu.edu.cn/mirLncRNA.php) [12], we found the putative complementary sequences for the seed region of *miR-340* on *SNHG14* gene (Figure 5A). To validate the direct binding between SNHG14 and *miR-340* at endogenous levels, dual luciferase reporter assay was thus performed. As shown in Figure 5B, cotransfection with pLUC-SNHG14-WT vector and *miR-340* mimics significantly reduced the luciferase activity in A549 cells. Next, we examined the levels of *miR-340* in A549 cells transfected with si-SNHG14 or pcDNA3.1-SNHG14, finding that SNHG14 knockdown increased, whereas SNHG14 overexpression decreased *miR-340* expression in A549 cells (Figure 5C). Meanwhile, the expression of *miR-340* in NSCLC and corresponding noncancerous tissues was also detected by RT-qPCR analysis. As expected, we found that *miR-340* is down-regulated in NSCLC tissues (Figure 5D), and more importantly, as exhibited in Figure 5E, there was a significantly inverse correlation between SNHG14 levels and *miR-340* levels in NSCLC tissues (*r* = −0.259, *P*=0.01). Collectively, these results strongly revealed a potential role of SNHG14 as a molecular sponge for *miR-340*.

**Figure 5:** SNHG14 acts as a sponge for *miR-340* in NSCLC cells (**A**) Predictive binding sites of *miR-340* on *SNHG14* gene. (**B**) Relative luciferase activity was analyzed in A549 cells cotransfected with pLUC-SNHG14-WT or pLUC-SNHG14-MUT and *miR-340* mimics or mimics control. (**C**) *miR-340* expression was determined by RT-qPCR analysis in A549 cells with SNHG14 overexpression or knockdown. Data were represented as the mean  ±  S.D. (**D**) *miR-340* expression was reduced in NSCLC tissues compared with the adjacent nontumor tissues. (**E**) The correlation between SNHG14 and *miR-340* levels in NSCLC tissues was evaluated by Pearson correlation analysis.

### *miR-340* restores the SNHG14-mediated NSCLC cell phenotypes

We then examined the effects of *miR-340* on SNHG14-mediated NSCLC cell phenotypes. *miR-340* mimics or mimics control was delivered into the A549 cells transfected with pcDNA3.1-SNHG14. As expected, SNHG14 overexpression induced increased cell proliferation, and enhanced cell cycle progression, was partially rescued by cotransfection of *miR-340* mimics (Figure 6A,B).

**Figure 6:** *miR-340* restores the SNHG14-mediated NSCLC cell phenotypes (**A**) Cell proliferation was determined by CCK-8 assay in A549 cells cotransfected with pcDNA3.1-SNHG14 and *miR-340* mimics. (**B**) Cell cycle distribution was determined by flow cytometer analysis in A549 cells cotransfected with pcDNA3.1-SNHG14 and *miR-340* mimics. Data were represented as the mean  ±  S.D. *P<0.05 compared with pcDNA3.1-SNHG14+miR-NC group.

## Discussion

NSCLC pathogenesis is a multistep process through the accumulation of genetic alterations. LncRNAs were previously considered to be simply transcriptional ‘noise’ or cloning artifacts [13]; however, in recent years, the importance of lncRNAs in NSCLC pathogenesis is gradually coming to light. Some lncRNAs act as tumor suppressors, while others act as tumor promoters. In the present study, we showed that SNHG14 expression is increased in NSCLC tissues and cell lines. We also found that *miR-340* is negatively regulated by SNHG14. Therefore, the data provided here support a molecular mechanism by which SNHG14 promotes tumorigenesis in NSCLC patients.

SNHG14 is frequently dysregulated in various types of human cancers. For example, Wang et al. [14] identified that SNHG14 was down-regulated in human glioma tissues and cell lines. However, the present study showed that in clinical NSCLC samples, SNHG14 was significantly up-regulated compared with the normal tissues, and increased SNHG14 expression is closely correlated with aggressive tumor progression and poor clinical outcome of NSCLC patients. Additionally, to support our clinical findings, we performed loss- and gain-of-function experiments *in vitro*. The results demonstrated that down-regulation of SNHG14 could remarkably inhibit NSCLC cell proliferation through inducing cell apoptosis and cell cycle arrest at G_0_/G_1_ phase, suggesting the oncogenic role of SNHG14 in NSCLC. Animal experiment also indicated that down-regulated SNHG14 greatly inhibited NSCLC tumor growth *in vivo*.

MiRNAs, a class of short (∼22 nts) non-coding RNAs, have been considered as critical regulators of cancer pathogenesis and progression [15]. Recent reports have described that lncRNAs might function as competing endogenous RNAs (ceRNAs) to regulate miRNAs and thus, in turn regulate the expression of specific genes targetted by miRNA [16]. For instance, SNHG12 promotes tumorigenesis and metastasis in hepatocellular carcinoma through acting as an endogenous sponge for *miR-199a/b-5p* [17]. With regard to *miR-340*, it has been widely reported as a tumor suppressive miRNA in many cancers, including NSCLC [18–20]. In the present study, we confirmed that SNHG14 might serve as an endogenous sponge that competes for binding to *miR-340* using dual luciferase reporter assay and the expression of *miR-340* was correlated negatively with the expression of SNHG14 in human NSCLC tissues.

In the present study, for the first time, we showed that SNHG14 expression is up-regulated in NSCLC tissues, and SNHG14 regulates apoptosis and proliferation of A549 cells via acting as a ceRNA for *miR-340* binding. Although more research needs to be done, the present findings will provide a new insight to explore the biology of this fatal disease.

## Abbreviations

ceRNA: competing endogenous RNA
lncRNA: long non-coding RNA
NSCLC: non-small cell lung cancer
OS: overall survival
si-NC: siRNA specifically targetting scrambled nucleotide
si-SNHG14: siRNA specifically targetting SNHG14
SNHG14: small nucleolar RNA host gene 14
